# Musical practice and BDNF plasma levels as a potential marker of synaptic plasticity: an instrument of rehabilitative processes

This article has been retracted.

**DOI:** 10.1007/s10072-020-04715-9

**Published:** 2020-09-17

**Authors:** Alessandro Minutillo, Gabriele Panza, Massimo Carlo Mauri

**Affiliations:** 1 Department of Neurosciences and Mental Health, Fondazione IRCCS Ca’ Granda Ospedale Maggiore Policlinico, Milan, Italy; 2 Department of Pathophysiology and Transplantation, University of Milan, Milan, Italy

**Keywords:** Psychiatric rehabilitation, Biological neurosciences, BDNF, Synaptic plasticity, Music

## Abstract

**Background and objectives:**

The aim of the study was to investigate the influence of musical practice on brain plasticity. BDNF (brain-derived neurotrophic factor) is a neurotrophin involved in neuroplasticity and synaptic function.

**Materials and methods:**

We recruited 48 healthy subjects of equal age and sex (21 musicians and 27 non-musicians). All subjects were administered the AQ (Autism-Spectrum Questionnaire) and plasma levels (PLs) of BDNF, oxytocin (OT), and vasopressin (VP) were measured in the blood sample of every participant.

**Results.:**

The difference between BDNF PLs in the two groups was found to be statistically significant (*t* = − 2.214, *p* = 0.03). Furthermore, oxytocin (OT) PLs and musical practice were found to be independent positive predictors of BDNF PLs (*p* < 0.04). We also found a negative correlation between BDNF PLs and AD (attention to detail) sub-scale score of AQ throughout the whole sample. Assuming BDNF PLs to be a marker of synaptic plasticity, higher PLs could be associated with the activation of alternative neural pathways: a lower score in the “attention to detail” sub-scale could imply greater flexibility of higher cerebral functions among musicians.

Further researches should be conducted to assess the rehabilitative usefulness of these findings among patients affected by psychiatric disorders.

## Introduction

In this study, we deal with the relationship between music and the brain. Music developed throughout human activities (becoming a crucial cultural aspect in every historical age), bearing interesting neurophysiological mechanisms. These ones underlie both listening and musical practice, and account for the evolutionary “success” of music, especially looking at its effects on the neural circuits of gratification [62]. Among the emotional responses elicited by music, pleasure is remarkably and intimately linked to the neural circuits of gratification (reward). The transition from perception to pleasure probably depends on a series of phenomena that connect the two [62]. The basis for these processes consists essentially of the following: temporal expectations, their associated forecasts, and the intensity of the reward generated by the satisfaction of these forecasts. The interactions between the cortical auditory regions and the frontal cortex (FC) are fundamental to allow the working memory to generate tonal and temporal expectations based on the structural regularities proper to music [33].

The satisfaction of the forecasts leads to a release of dopamine in the striatum (nucleus accumbens, NAcc), a response that is further intensified when the reward is better than expected.

The interaction between the auditory cortices and the striatum demonstrates the existence of an intense communication between structures of analysis/pattern processing (cortical) and reward systems (subcortical).

Some aspects about cellular neurobiology are crucial when trying to understand how the human brain is able to adapt to learning music. The term “brain plasticity” generally describes the brain adaptation of a sensory or a motor system to environmental stimuli and functional requests, or the compensation of damaged structures [6, 12, 18, 23, 25, 29, 37–40, 43, 44, 47–49, 51, 52, 59, 62, 65].

These neurobiological aspects can be important to explain the increased brain plasticity found in musicians by many neuroimaging studies [50]. On the other hand, these evidences might be considered the biological basis of clinical and rehabilitative implications investigated by numerous studies on music intervention (MI) programs (interactive or passive, like singing songs, instrumental improvisations, and listening music tracks) which showed the effectiveness of MI in cognitive, mood, and behavior disorders [17, 36, 57].

In our study, we investigated if these adaptations can reflect functional differences between musicians and non-musicians [50] focusing on an important neurotrophic factor involved in synaptic plasticity, the brain-derived neurotrophic factor (BDNF).

BDNF is a 14-kDa protein that, in humans, is encoded by the BDNF gene, located on the short arm of chromosome 11 (11p14.1) [27, 34, 46, 56]. Like all neurotrophic factors, it is found in both the central and peripheral nervous systems.

There are multiple mechanisms by which neuronal activity can increase the specific expression of BDNF; one of these, is the activation of NMDA postsynaptic receptor and then the activation of a biosignal pathway mediated by the Erk, CaM KII/IV, PI3K, and PLC proteins, which is able to start the transcription of BDNF [63].

BDNF is released from the postsynaptic membrane in an activity-dependent way, as it acts on local TrkB receptors [32].

Furthermore, the activation of the D5 dopamine receptor promotes the expression of BDNF in the prefrontal cortex [42].

Among the single-nucleotide polymorphisms (SNPs) of its gene, the Val66Met is probably the most studied, since it is able to influence in a rather significant way the structure and the function of the central nervous system [5, 15].

BDNF acts on some neurons of the nervous system, increasing their survival and stimulating the generation, growth, and differentiation of new neurons and synapses [1, 7, 8, 11, 19, 21, 22, 24, 35, 41, 53–55, 60, 64].

This study examined plasma levels (PLs) of BDNF (brain-derived neurotrophic factor), oxytocin (OT), and vasopressin (VP) in musicians and compared them with controls of equal age and sex. Furthermore, every participant was administered the Autism-Spectrum Questionnaire (AQ).

## Study aim

The study aims to evaluate the possible correlation between the neurobiochemical variables BDNF, OT, and VP PLs and musical practice; this could help to understand the neurobiological differences between musicians and the general population, in terms of synaptic brain plasticity, in the light of the rehabilitative efficacy of music therapy in neuropsychiatric disorders.

## Materials and methods

A case-control study was designed recruiting 48 healthy subjects: 21 musicians and 27 non-musicians. To be defined as a “musician,” the practice of any musical instrument or voice was required for at least 3 h a week. This practice had to be stable and continued for at least 5 years and the subject had to have been achieved a musical degree.

An informed consent was obtained from each participant and the research was conducted according to the principles of the Helsinki Declaration.

### Inclusion criteria

Being a musician, defined as follows:

• Practice of any musical instrument or voice for at least 3 h a week.

• The musical practice had to be stable and continued for at least 5 years.

• The subject had to own a musical degree in a specific instrument.

### Exclusion criteria

• Age < 18 years.

• Presence of major internal or surgical diseases.

• Presence of psychiatric disorders.

• Presence of allergic diathesis.

• For female subjects: pregnancy.

### Assessment

After the recruitment, everyone was asked to complete the AQ (Autism-Spectrum Quotient) questionnaire and to provide a blood sample. The biological sample was taken at 10:00 am (in order to minimize a potential circadian rhythm) from the antecubital vein and stored in a vacutainer tube. The blood was immediately centrifuged at 1000*g* for 15 min and the plasma obtained was aliquoted and stored at − 20 °C until analysis. BDNF, OT, and VP PLs were dosed using an ELISA method (enzyme-linked immunosorbent assay) (R&D Systems, Inc. Minneapolis, MN) according to the manufacturer’s instructions.

### Autism-Spectrum Quotient

The Autism-Spectrum Quotient (AQ) is a questionnaire developed by Baron-Cohen and colleagues [3], and consists of a rapid and self-administered clinical tool designed to measure where a normal-IQ adult is placed in the continuum of autistic socio-communicative disability, that is, how much he or she presents “autistic traits” or, as defined by Bailey [2], the “extended phenotype.” Anyway, the AQ represents only a screening test and not a real diagnostic tool.

It is made up by 50 questions divided into 5 sub-groups of 10 questions each, which evaluate 5 different areas of ability: social skills (SS), attention switching (AS), attention to details (AD), communication (C), and imagination (I). According to the indications of Baron-Cohen [3], the cut-off which distinguishes individuals with clinical levels of potentially significant autistic traits is a score of 32.

### Oxytocin and vasopressin

Oxytocin (OT) and vasopressin (VP or ADH, antidiuretic hormone) are two nona-peptides produced mainly by the supraoptic and paraventricular nuclei of the hypothalamus. OT plays an important “pro-social” role, favoring empathy and “mind-reading,” probably leading to an increase in the salience of social stimuli. Studies conducted in humans showed that exogenous administration of oxytocin increases confidence towards other people [31], generosity [61], empathy [4], and altruism [13]. Moreover, both OT and VP facilitate sexual and parenting behaviors in mammals: OT promotes sexual relations, maternal attachment to the newborn, and pair bond [9]. In contrast, VP mediates typically male behaviors such as aggression and territoriality; moreover, it seems to play an important role in memory and anxiety [20].

### Statistical analysis

A descriptive statistic has been calculated for all the variables. The normally distributed variables were presented as mean and standard deviation (SD); the variables not normally distributed were presented as medians and interquartile ranges, while the categorical variables were expressed as raw numbers and percentages. The differences between the two groups at the baseline were evaluated by the Student's *t* test. The correlations between variables were evaluated by the Pearson coefficient. A multivariate linear regression model was used, using BDNF PLs as a dependent variable and sex, musical practice, total AQ, VP PLs, and OT PLs as independent predictors. A two-tailed *p* value < 0.05 was considered statistically significant. All analyses were performed using the SPSS 20.0 software.

## Results

The general characteristics of our sample and their mean results ± SD in the total AQ and its sub-scales are shown in Table 1. The subjects were mostly young adults and both genders were equally represented.

**Table 1:** Age, sex, and mean ± SD of AQ results of the sample studied

	Musicians (*n* = 21)	Non-musicians (*n* = 27)	*p* value
Age (years*)*	47.20 ± 24.45	55.30 ± 37.63	ns
Sex (%)			ns
Male	56.5% (12)	44.4% (12)	
Female	43.6% (9)	55.6% (15)	
AQ (total)	15.43 ± 6.00	16.59 ± 5.68	ns
AD (attention to detail)	4.73 ± 2.14	5.81 ± 1.92	ns
AS (attention switching)	4.32 ± 2.38	4.27 ± 1.40	ns
C (communication)	2.32 ± 1.84	2.00 ± 1.60	ns
I (imagination)	2.23 ± 1.44	2.42 ± 1.77	ns
SS (social skills)	2.05 ± 1.46	2.00 ± 2.12	ns
Vasopressin (pg/mL)	45.59 ± 18.96	54.53 ± 34.60	ns
BDNF (ng/mL)	9.72 ± 11.73	3.98 ± 2.09	0.03
Oxytocin (pg/mL)	524.61 ± 279.09	542.25 ± 285.08	ns

The age was not statistically different between the two groups (*t* = 0.082, *p* = 0.93). Similarly, the gender of the participants was also uniformly distributed.

Taking into account the AQ scores and its sub-scales, no statistically significant differences were found between the two groups (total AQ: *t* = 0.70, *p* = 0.487; AD: *t* = 1.843, *p* = 0.072; AS: *t* = − 0.085, *p* = 0.93; C: *t* = − 0.642, *p* = 0.524; I: *t* = 0.415, *p* = 0.68; SS: *t* = − 0.085, *p* = 0.93).

Looking at biochemical parameters, the difference in VP PLs was not statistically significant in the two groups (*t* = 1.132, *p* = 0.264). A similar result was found for OT PLs (*t* = 1.177, *p* = 0.861).

BDNF PLs were statistically different in the two groups (*t* = − 2.214, *p* = 0.03), as also reported in the graph showed in Fig. 1.

**Fig. 1:** Comparison between musicians and non-musicians: mean BDNF plasma levels (*p* < 0.05)

Observing the correlations existing between the various parameters, there was a statistically significant negative relationship between BDNF PLs and the AD sub-scale (*r* = − 0.30, *p* = 0.04) (Fig. 2).

**Fig. 2:** Correlation between BDNF plasma levels and results in the AD sub-scale of AQ (Autism-Spectrum Quotient) (*p* < 0.05)

Using a multivariate linear regression with BDNF PLs as a dependent variable and sex, musical practice, total AQ, VP PLs, and OT PLs as independent predictors, the resulting model (*p* = 0.011) was able to explain 48% of the variance of the dependent variable. The only significant predictors were musical practice (*p* = 0.05) and OT PLs (*p* = 0.02) (Table 2).

**Table 2:** Multivariate linear regression model between BDNF PLs and sex, musical practice, total AQ, vasopressin PLs, and oxytocin PLs as independent predictors

Variable	*b*	*β*	*p* value
Sex	− 0.730	− 0.114	0.485
Musical practice	2.112	0.331	0.05*
AQ (total)	0.124	0.239	0.158
*Vasopressin (pg/mL)*	− 0.012	− 0.104	0.529
*Oxytocin (pg/mL)*	− 0.006	− 0.548	0.002*

*R*^2^ = 0.483, adjusted *R*^2^ = 0.360

*p* = 0.011

*p ≤ 0.05

*AQ*, Autism-Spectrum Quotient

## Discussion

Our study showed higher BDNF PLs in musicians compared with control of the same age and gender. Furthermore, OT PLs and musical practice were found to be independent positive predictors of BDNF PLs.

Given that there is a direct relationship between BDNF PLs and its concentrations in the central nervous system [30], it could be hypothesized that higher PLs in musicians correspond to higher concentrations in their brain. This data could provide a neurobiochemical explanation to the increased brain plasticity found in musicians by many neuroimaging studies [50].

The clinical and rehabilitative implications of this phenomenon have been investigated by numerous studies, since a broad spectrum of music intervention (MI) programs (interactive or passive) are known: singing songs of the repertoire of light and popular music, music/movement associations, instrumental improvisation and listening to music tracks, and showing the effectiveness of MI in cognitive, mood, and behavior disorders [17, 36, 57]. Functional magnetic resonance imaging (fMRI) studies conducted during music rehabilitative interventions (e.g., music listening) have shown connectivity modifications in different brain networks, enhancing also cognitive and mood aspects: memory, attention, executive functions, and depression [28, 45]. In schizophrenia or schizophrenia-like disorders, some evidences suggest that music therapy as an addition to standard care can improve the global state, mental state (including negative and general symptoms), social functioning, and quality of life. On the other hand, effects seem to depend on the number of music therapy sessions as well as the quality of the music therapy provided [16]. In dementia, music listening coupled with cognitive elements (reminiscence and attention training) showed to improve overall cognitive performances and neuropsychiatric symptoms versus the standard care [58]. Furthermore, a randomized controlled study showed that music therapy, added to pharmacological treatment in adult psychiatric patients (affected by schizophrenia, bipolar disorder, schizoaffective disorder, major depressive disorder, or specific personality disorder), determined a significantly greater reduction in neuroleptic dosage among the participants who received group music therapy versus the control group [14].

In the present study, we also observed an inverse correlation between BDNF PLs and AD (attention to detail) scores in the whole sample: this could furtherly suggest a close link among BDNF, synaptic plasticity, and cognitive processes. In fact, a greater synaptic plasticity, expressed by higher BDNF PLs, could establish alternative neural pathways, with a consequent lower rigidity of the cognitive functioning [26]: a lower score in the AD sub-scale could be interpreted as an index of greater flexibility of the higher order brain capacities.

The study bears some limitations to consider before interpreting the results. First of all, its design does not allow to draw causal conclusions about the observed variables. For this purpose, a prospective study with multiple determinations of BDNF PLs in musicians and controls may be able to better clarify the observed relationship. Moreover, our sample is not large enough and consists mainly of young subjects. Future researches will be necessary in order to corroborate the results obtained, with larger sample sizes and a broader age range. Finally, we cannot state BDNF PLs to be a consequence of practice alone and not also of music listening: our control group, although not composed by music lovers, presented a minimum of listening activity which was difficult to quantify.

Therefore, it is possible to consider a future study which could analyze, in addition to musical practice, also the intensity of music listening, comparing three groups: poor musical listening, high musical listening, and listening and musical practice together. On the other hand, the BDNF PLs measured before and after a MI program could be used as a potential biological marker of the outcome, of course, combined with the clinical evaluation.

We believe that music is a fundamental constituent in every area of ​the anthropological sphere, so much that it is also used for experimental and hopefully ever more rehabilitative purposes in many neuropsychiatric conditions [10].
